The article "Analysis of Serum Interleukin-37 Level and Prognosis in Patients with ACS" was published in 2021. Journal: Comput Math Methods Med.

# Analysis of Serum Interleukin-37 Level and Prognosis in Patients with ACS

**DOI:** 10.1155/2021/3755458

**Published:** 2021-09-17

**Authors:** Canjun Liu, Yancui Cui, Dan Zhang, Xiao Tian, Hongyan Zhang

**Affiliations:** ^1^Department of No. 2 Cardiology, The Third Affiliated Hospital of Qiqihar Medical University, China; ^2^Department of No. 5 Cardiology, The Third Affiliated Hospital of Qiqihar Medical University, China

## Abstract

**Objective:**

To explore the level of serum interleukin-37 in patients with acute coronary syndrome (ACS) and its prognostic value.

**Methods:**

Altogether, 121 continuous ACS cases from September 2017 to June 2020 were selected as the research group (RG), and 107 healthy individuals during the same period were obtained as the control group (CG). ELISA was applied to test IL-37 in the serum of the CG and the RG. Chemiluminescence immunoassay was applied to test NT-pro BNP and hs-cTnI in each group and immune scattering turbidimetry to test hs-CRP. The correlation of IL-37 with serum NT-pro BNP, hs-cTnI, and CRP was analyzed, and the value of IL-37 in diagnosis and prognosis prediction of patients with ACS was tested. Logistic regression was applied to test the independent risk factors affecting poor prognosis of patients with ACS.

**Results:**

IL-37 was poorly expressed in patients with ACS, which had a high diagnostic value for ACS (sensitivity: 94.39%, specificity: 74.38%, and area under curve: 0.945). There was a negative correlation of IL-37 with serum NT-pro BNP, hs-cTnI, and CRP. IL-37 in patients with poor prognosis was markedly declined compared with that of patients with good prognosis, and the predicted AUC was 0.965. Logistic regression revealed that low IL-37, diabetes, high CRP, NT-pro BNP, and hs-cTnI in the blood were independent risk factors for poor prognosis in patients with ACS.

**Conclusion:**

IL-37 is low expressed in patients with ACS, which has a good diagnostic and prognostic value for ACS, and may be applied as an important marker for the prediction of patients with ACS.

## 1. Introduction

Acute coronary syndrome (ACS) is a common critical illness of cardiovascular system. With the development of medical technology, patients with ACS have been treated in a standardized and timely manner to a great extent, which has achieved good results [1, 2]. The short-term effect is good, but the long-term prognosis of ACS is still not optimistic [3]. In the follow-up rehabilitation after discharge, many patients are often faced with readmission due to adverse cardiovascular events [4]. Therefore, finding a reliable marker to evaluate and predict the prognosis of patients is of great significance for timely adjusting the follow-up rehabilitation plan of patients and reducing the occurrence of adverse cardiovascular events.

Interleukin-37 (IL-37) is a new factor with homologous DNA of IL-1 family found in 2000 [5]. However, unlike other IL family members, IL-37, a newly discovered anti-inflammatory cytokine, is a natural innate immunosuppressant, which has potential protective effects in inflammatory bowel disease, hepatic ischemia reperfusion, and other diseases [6, 7]. In recent years, some studies have found that IL-37 might be closely correlated to the growth of atherosclerosis and that IL-37 may inhibit the release of inflammatory factors in atherosclerosis through MAPK inflammatory signaling pathway and inflammatory mediators [8, 9]. Although previous studies [10] found that there were some differences in IL-37 in patients with ACS, the specific correlation of IL-37 with ACS and the prediction of patients' prognosis have not been discussed yet.

Therefore, in this research, IL-37 in local plasma of patients with ACS was tested and the occurrence of adverse events of patients was followed up for 3 months, so as to test the function of IL-37 in the progression of ACS.

## 2. Materials and Methods

### 2.1. Clinical Data

Altogether 121 continuous ACS cases from September 2017 to June 2020 were obtained as the research group (RG), including 63 males and 58 females with an average age of 67.89 ± 5.52 years, 107 healthy individuals during the same period were obtained as the control group (CG). The patients in the RG all met the diagnostic criteria of ACS [11]. Those with other malignant tumor diseases, severe hepatic or renal insufficiency, other serious endocrine diseases, and other acute and chronic inflammation-related diseases or those who did not cooperate with the research were excluded. The informed consent forms were obtained from the patients. This research conformed to the Ethics Committee and the Declaration of Helsinki.

### 2.2. Index Detection

IL-37 in serum of two groups was tested using ELISA. The kit was obtained from Beijing Bio Friend and produced by R&D systems (US), and the operation was strictly in accordance with the product instructions. NT-pro BNP and hs-cTnI in the CG and the RG were tested using chemiluminescence immunoassay analyzer (the instrument was chemiluminescence immunoassay analyzer from Abbott, and the kit was the original reagent). hs-CRP was tested using immunonephelometry.

### 2.3. Prognostic Assessment

According to the occurrence of cardiovascular events (including repeated ischemic angina attacks, new or worsening cardiac insufficiency, severe arrhythmia, and death) within 30 days after admission, patients with one or more cardiovascular events within 30 days after admission were classified as the cardiovascular event group, while patients without cardiovascular event were the noncardiovascular event group.

### 2.4. Statistical Method

SPSS20.0 (Bizinsight, Beijing, CN) was applied for the statistical analysis of experimental data. A chi-square test was applied for counting data, and the measurement data were represented as the mean ± SD. A *t*-test was applied for pair-wise comparison, a paired *t*-test for comparison before and after intervention, Pearson's test for correlation analysis, and GraphPad Prism 6 for visualizing the experimental pictures. When *P* < 0.05, there were statistical differences.

## 3. Result

### 3.1. General Information

There was no remarkable difference in sex, age, BMI, and smoking history (*P* > 0.05), which is comparable (Table 1).

### 3.2. Il-37 in Patients with ACS and Its Diagnostic Value

IL-37 in the RG was markedly lower than that in the CG (*P* < 0.05). ROC curve analysis showed that IL-37 had high sensitivity (94.39%) and specificity (74.38%), and its AUC was 0.945 (Figure 1).

### 3.3. Comparison of Other Related Indexes

NT-pro BNP, hs-cTnI, and CRP in the RG were markedly elevated compared with those in the CG (*P* < 0.05) (Table 2).

### 3.4. Correlation Analysis of IL-37 with NT-pro BNP, hs-cTnI, and CRP

The correlation of IL-37 with NT-pro BNP, hs-cTnI, and CRP in patients with ACS was tested. The results revealed that IL-37 was negatively correlated with these indicators (*P* < 0.001) (Figure 2).

### 3.5. Correlation of IL-37 with the Prognosis

The individuals were grouped into the cardiovascular event group (62 cases) and noncardiovascular event group (59 cases) according the occurrence of adverse cardiovascular events. By comparing IL-37 in patients with cardiovascular events, we found that IL-37 in the cardiovascular event group was markedly declined compared with that in the noncardiovascular event group (*P* < 0.05), and the ROC curve showed that IL-37 had a high predictive value for cardiovascular events in patients with ACS (sensitivity: 96.61%) (Figure 3).

### 3.6. Univariate Analysis of Poor Prognosis of Patients

In order to further test the various factors affecting the prognosis of ACS, a univariate analysis was conducted. The results revealed that the prognosis was related to diabetes mellitus, CRP, NT-pro BNP, and hs-cTnI levels (all *P* < 0.05 or *P* < 0.01) (Table 3).

### 3.7. Multivariate Analysis of Poor Prognosis in Patients with ACS

The low IL-37, diabetes mellitus, high CRP, NT-pro BNP, and hs-cTnI in the blood were included in the analysis, and the occurrence of cardiovascular events was taken as the dependent variable. The logistic regression model was applied for multivariate analysis. The results revealed that the low IL-37, diabetes mellitus, high CRP, NT-pro BNP, and hs-cTnI were independent risk markers for poor prognosis (Table 4).

## 4. Discussion

At present, the basic pathophysiological mechanism of ACS is inflammatory reaction. In the past, the inflammatory mediators involved in ACS mainly included CRP, IL-6, and other factors [12, 13]. However, with the deepening of medical research, it has been found that IL-37 is also an inflammatory factor related to ACS [14].

IL-37, a member of the IL-1 group, has an anti-inflammatory effect. In vivo and in vitro experiments suggested that IL-37 binds to TLR receptor-2 or TLR receptor-4 on the cell surface, inhibits the activation of NF-*κ*B, inhibits the production of monocyte chemotactic protein 1 (MCP1) and monocyte aggregation, promotes the secretion of TGF-*β*, alleviates inflammatory reaction, and improves myocardial ischemia and left ventricular function [15]. At present, there are relatively few reports about the role IL-37 in ACS. In order to find new possible indicators for the diagnosis and prognosis of patients with ACS, IL-37 in ACS cases and its related role were tested. Firstly, IL-37 in ACS cases and its diagnostic value were explored. The results revealed that IL-37 declined markedly. ROC curve indicated that IL-37 had good diagnostic effect for ACS. However, there are some controversies about the content of IL-37 in ACS cases. For example, some studies [16] found that IL-37 in severe coronary artery calcification elevated markedly. Other studies [17] found that IL-37 in coronary artery stenosis was markedly declined, which was consistent with our observation. The research also pointed out that the main effect of IL-37 was to reduce excessive inflammatory reaction through negative feedback, which played a very important role in the innate and adaptive immune system [18]. In addition [19], IL-37 reduced the area ratio of aortic plaque to vascular lumen markedly. IL-37 inhibited the induction of M1 macrophages induced by ox-LDL from peripheral monocytes and promoted the transformation of macrophages into M2 cells. These indicated that IL-37 can prevent atherosclerosis by regulating the polarity of macrophages. This further confirmed the role of IL-37 in ACS.

Then, in order to further test the clinical significance of IL-37 in ACS, the contents of NT-pro BNP, hs-cTnI, and CRR of patients were tested, and their correlation with IL-37 was confirmed. hs-cTnI is an important index for testing myocardial contractility, and it has obvious regulation effect on myocardial contraction [20]. NT-pro BNP, a member of natriuretic peptide cluster, has diuretic, vasodilating, and sympathetic nerve inhibiting effects. The research [21] showed that NT-pro BNP is mainly secreted by left ventricular myocytes, and it is relatively sensitive to changes in ventricular wall tension and ventricular load, and its expression level can reflect the severity of myocardial injury. NT-pro BNP, hs-cTnI, and CRP in ACS cases were markedly increased, and these indicators had a negative correlation with IL-37, which also suggested that IL-37 acts in myocardial contraction and myocardial injury. Then, we also explored the correlation of IL-37 with the prognosis of patients. The results revealed that IL-37 of patients with better prognosis was markedly higher than that of patients with poor prognosis, and ROC curve analysis showed that IL-37 had a good predictive value for poor prognosis of patients with ACS. At present, since the discovery of IL-37, its anti-inflammatory, and cardioprotective mechanism has not been completely determined, its anti-inflammatory, immunomodulatory, and metabolic activities have been confirmed [22]. These mechanisms have an important impact on the prognosis of patients with ACS. Finally, in order to further explore the factors affecting the prognosis of ACS cases, a logistic regression test was conducted. The low IL-37, diabetes mellitus, high CRP, NT-pro BNP, and hs-cTnI were independent risk factors affecting poor prognosis of patients with ACS. This indicated that if the patients' IL-37, CRP, NT-pro BNP, hs-cTnI, and diabetes can be well controlled, the prognosis of patients can also be improved.

There are also some limitations in our manuscript. First, the retrospective nature of the study may bring some bias to the results. Second, the aim of the study is to explore the diagnostic and prognostic values of IL-37 for ACS patients; thus, the other markers CRP, NT-pro BNP, and hs-cTnI could not be studied in depth.

To sum up, the low IL-37 in serum of patients with ACS has a good diagnostic and prognostic value for ACS, and it is an independent risk marker for poor prognosis of ACS cases, which may be applied for diagnosis and prognosis prediction of ACS.

## Figures and Tables

**Figure 1:** IL-37 in patients with ACS and its diagnostic value. (a) IL-37 in patients with ACS; (b) ROC curve analysis of IL-37 on ACS. ∗ indicates *P* < 0.05.

**Figure 2:** Correlation analysis of IL-37 with NT-pro BNP, hs-cTnI, and CRP. (a) Correlation analysis of IL-37 with NT-pro BNP; (b) correlation analysis of IL-37 with hs-cTnI; (c) correlation analysis of IL-37 with CRP.

**Figure 3:** Correlation of IL-37 with prognosis of patients. (a) IL-37 in patients with different prognosis; (b) IL-37 can predict the poor prognosis of patients with ACS. ∗ indicates *P* < 0.05.

**Table 1:** General information.

Factors	RG (*n* = 121)	CG (*n* = 107)	*t*/*X*^2^	*P*
Gender			0.010	0.920
Male	63 (52.07)	55 (51.40)		
Female	58 (47.93)	52 (48.60)		
Age (years)	67.26 ± 5.28	67.31 ± 5.31	0.071	0.943
BMI (kg/m^2^)	23.05 ± 1.24	23.14 ± 2.26	0.378	0.706
Drinking history			0.184	0.668
Yes	77 (63.64)	71 (66.36)		
No	44 (36.36)	36 (33.64)		
Smoking history			0.232	0.630
Yes	64 (52.89)	60 (56.07)		
No	57 (47.11)	47 (43.93)		
Disease type			—	—
Unstable angina pectoris	42 (34.71)	—		
ST-segment elevation myocardial infarction	37 (30.58)	—		
Non-ST segment elevation myocardial infarction	42 (34.71)	—		
Serum uric acid (mmol/L)	265.71 ± 21.75	263.84 ± 20.49	0.666	0.506
Hemoglobin (g/L)	138.75 ± 2.58	138.46 ± 2.61	0.842	0.400

**Table 2:** Comparison of other related indexes.

Factors	RG (*n* = 121)	CG (*n* = 107)	*t*	*P*
NT-pro BNP (pg/mL)	268.39 ± 22.49	45.13 ± 4.79	100.7	<0.001
hs-cTnI (ng/mL)	0.72 ± 0.08	0.01 ± 0.00	91.78	<0.001
CRP (mg/L)	9.34 ± 1.22	1.14 ± 0.13	69.16	<0.001

**Table 3:** Univariate analysis of poor prognosis of patients.

Factors			*χ* ^2^	*P*
	Cardiovascular event group (*n* = 62)	No cardiovascular event group (*n* = 59)		
Age			0.002	0.961
≥67 years	36 (58.06)	34 (57.63)		
<67 years	26 (41.94)	25 (42.37)		
Gender			0.069	0.794
Male	33 (51.92)	30 (48.98)		
Female	29 (48.08)	29 (51.02)		
Complicated with diabetes			18.20	<0.001
Yes	45 (72.58)	20 (33.90)		
No	17 (27.42)	39 (66.10)		
NT-pro BNP (pg/mL)	435.19 ± 33.27	405.61 ± 27.49	7.262	<0.001
hs-cTnI (ng/mL)	0.89 ± 0.22	0.75 ± 0.18	5.217	
CRP (mg/L)	10.24 ± 2.36	8.27 ± 1.19	7.801	
Serum creatinine (*μ*mmol/L)	76.49 ± 3.28	77.05 ± 3.11	1.318	0.189
Hemoglobin (g/L)	136.49 ± 3.18	137.11 ± 3.21	1.463	0.145

**Table 4:** Multivariate analysis of poor prognosis in patients with coronary heart disease.

Factors	*β*	SE	Wald	OR	95% CI	*P*
IL-37	0.455	0.217	4.664	1.631	1.031~2.412	0.012
Diabetes	0.887	0.379	6.113	2.542	1.672~3.593	<0.001
Blood CRP	0.675	0.284	5.211	1.949	1.097~3.474	0.015
NT-pro BNP	0.623	0.308	4.428	1.894	1.041~3.405	0.032
hs-cTnI	1.061	0.485	5.254	2.991	1.173~7.522	<0.001

## Data Availability

All the raw data could be accessed by contacting the corresponding author if needed.

## References

[1] Montenegro Sa F., Carvalho R., Ruivo C. (2019). Beta-blockers for post-acute coronary syndrome mid-range ejection fraction: a nationwide retrospective study. *European Heart Journal Acute Cardiovascular Care*.

[2] Deharo P., Cuisset T. (2020). Optimal duration of dual antiplatelet therapy post percutaneous coronary intervention in acute coronary syndrome. *Trends in Cardiovascular Medicine*.

[3] Soria-Florido M. T., Castañer O., Lassale C. (2020). Dysfunctional high-density lipoproteins are associated with a greater incidence of acute coronary syndrome in a population at high cardiovascular risk: a nested case-control study. *Circulation*.

[4] Pocock S. J., Huo Y., Van de Werf F. (2019). Predicting two-year mortality from discharge after acute coronary syndrome: an internationally-based risk score. *European Heart Journal Acute Cardiovascular Care*.

[5] Kumar S., McDonnell P. C., Lehr R. (2000). Identification and initial characterization of four novel members of the interleukin-1 family. *The Journal of Biological Chemistry*.

[6] Tetè S., Tripodi D., Rosati M. (2012). IL-37 (IL-1F7) the newest anti-inflammatory cytokine which suppresses immune responses and inflammation. *International Journal of Immunopathology and Pharmacology*.

[7] Sakai N., Van Sweringen H. L., Belizaire R. M. (2012). Interleukin-37 reduces liver inflammatory injury via effects on hepatocytes and non-parenchymal cells. *Journal of Gastroenterology and Hepatology*.

[8] Wu B. W., Zeng Q. T., Meng K., Ji Q. W. (2013). The potential role of IL-37 in atherosclerosis. *Pharmazie*.

[9] Wong C. K., Cheung P. F., Ip W. K., Lam C. W. (2005). Interleukin-25-induced chemokines and interleukin-6 release from eosinophils is mediated by p38 mitogen-activated protein kinase, c-Jun N-terminal kinase, and nuclear factor-*κ*B. *American Journal of Respiratory Cell and Molecular Biology*.

[10] Liu K., Tang Q., Zhu X., Yang X. (2017). IL-37 increased in patients with acute coronary syndrome and associated with a worse clinical outcome after ST-segment elevation acute myocardial infarction. *Clinica Chimica Acta*.

[11] Mao X., Zhu R., Zhang F. (2019). IL-37 plays a beneficial role in patients with acute coronary syndrome. *Mediators of Inflammation*.

[12] Shuvy M., Beeri G., Klein E. (2018). Accuracy of the Global Registry of Acute Coronary Events (GRACE) risk score in contemporary treatment of patients with acute coronary syndrome. *The Canadian Journal of Cardiology*.

[13] Kim S. W., Kang H. J., Bae K. Y. (2018). Interactions between pro-inflammatory cytokines and statins on depression in patients with acute coronary syndrome. *Progress in Neuro-Psychopharmacology and Biological Psychiatry*.

[14] Al Shahi H., Shimada K., Miyauchi K. (2015). Elevated circulating levels of inflammatory markers in patients with acute coronary syndrome. *International Journal of Vascular Medicine*.

[15] Yousif N., Li J., Yousif F. (2011). Expression of IL-37 in mouse protects themyocardium against ischemic injury via modulation of NF-*κ*B activation. *Circulation*.

[16] Chai M., Zhang H. T., Zhou Y. J. (2017). Elevated IL-37 levels in the plasma of patients with severe coronary artery calcification. *Journal of Geriatric Cardiology*.

[17] Liu T., Han C., Sun L. (2019). Association between new circulating proinflammatory and anti-inflammatory adipocytokines with coronary artery disease. *Coronary Artery Disease*.

[18] Gao W., Kumar S., Lotze M. T., Hanning C., Robbins P. D., Gambotto A. (2003). Innate immunity mediated by the cytokine IL-1 homologue 4 (IL-1H4/IL-1F7) induces IL-12-dependent adaptive and profound antitumor immunity. *Journal of Immunology*.

[19] Huang J., Hou F. L., Zhang A. Y., Li Z. L. (2016). Protective effect of the polarity of macrophages regulated by IL-37 on atherosclerosis. *Genetics and Molecular Research*.

[20] Kimenai D. M., Lindahl B., Jernberg T., Bekers O., Meex S. J. R., Eggers K. M. (2020). Sex-specific effects of implementing a high-sensitivity troponin I assay in patients with suspected acute coronary syndrome: results from SWEDEHEART registry. *Scientific Reports*.

[21] Guo G., Huang Z., Wang S., Chen X. (2020). Sex differences in uric acid and NT-pro BNP assessments during coronary severity. *Medicine (Baltimore)*.

[22] Lopez-Bautista F., Posadas-Sanchez R., Vazquez-Vazquez C., Fragoso J. M., Rodriguez-Perez J. M., Vargas-Alarcon G. (2020). IL-37 gene and cholesterol metabolism: association of polymorphisms with the presence of hypercholesterolemia and cardiovascular risk factors. The GEA Mexican Study. *The GEA Mexican Study. Biomolecules*.

